# Clinical Evaluation of Levetiracetam in the Treatment of Epilepsy

**DOI:** 10.1155/2022/3789516

**Published:** 2022-04-05

**Authors:** Haohao Wu, Jia Liu, Fang Qian, Junsu Yang, Yue Wang, Shaoyong Guan

**Affiliations:** ^1^Department of Neurology, Qujing First People's Hospital, Yunnan, Qujing 650000, China; ^2^Department of Pediatric Medicine, Qujing First People's Hospital, Yunnan, Qujing 650000, China

## Abstract

**Objectives:**

Epilepsy is a chronic neurological disorder that is characterized by episodes of seizure.

**Methods:**

In this study, patients with status epilepticus in the Intensive Care Unit of the Department of Neurology of Qujing First People's Hospital were collected and treated with levetiracetam injection, continuous bedside EEG monitoring (cEEG) technology, and quantitative EEG (qEEG) technique. The inhibitory effects of different doses of levetiracetam injection and sodium valproate on abnormal discharge, the improvement of clinical symptoms, the incidence of adverse reactions, and prognosis were monitored, analyzed, and compared.

**Results:**

Compared with the experimental group of sodium valproate, 1000 mg/d levetiracetam group and 1500 mg/d levetiracetam group had a high probability of successful symptom control and a short control time. The patients had a low recurrence rate and a long recurrence time, and the probability of abnormal discharge in EEG was low.

**Conclusions:**

The recording results showed that levetiracetam could significantly inhibit the abnormal discharge of patients. Compared with sodium valproate, high-dose levetiracetam is a drug with a rapid effect, good effect, and long action time.

## 1. Introduction

Status epilepticus (SE) is traditionally defined as one seizure lasting more than 30 minutes or repeated seizures lasting more than 30 minutes, and there is no recovery of consciousness between seizures. Refractory status epilepticus (RSE) refers to the acute, critical, and severe patients whose seizure time is more than 1 hour when the second-line drugs are ineffective [1]. However, when the duration of any type is >30 minutes (T2), it will lead to long-term adverse consequences such as neuronal death, neuronal injury, and neuronal network change [2]. Therefore, on the basis of controlling the primary disease, safely and quickly terminating the attack and restoring the patient's consciousness is an important means to save the patient's life and reduce the sequelae. Some investigations show that the incidence of SE is about 17–23 times per 100000 people [3], and 10%–40% of SE patients will develop RSE [4]. The mortality rate of patients is 16%–43.5% [5]. In the past, the primary treatment measure for early SE (T1) was benzodiazepines, but the overall control rate was not high (59–65%) [6]. At this time, second-line drugs were needed to control the attack, but the second-line drugs commonly used in China (phenytoin sodium, phenobarbital, and sodium valproate) had side effects of different degrees [7] (FDA: grade D), which increases the burden of patients and workload of doctors, and the dosage range is relatively limited. For the third-line drugs for the treatment of RSE, anesthetic agents (propofol and midazolam) need to be carried out with the aid of the endotracheal intubation ventilator, which will increase the pain and medical expenses of patients and may lead to poor prognosis. Therefore, how to quickly and effectively control status epilepticus and try to avoid adverse reactions has always been a thorny problem for doctors.

The occurrence of SE/RSE is usually accompanied by other serious brain diseases, such as central nervous system infection, hypoxic encephalopathy after CPR, CJD, and other serious metabolic/toxic encephalopathy. These patients have complicated conditions, and it is particularly difficult to treat patients with PEDs, with poor prognosis [8]. On the basis of actively controlling the primary disease, how to quickly and effectively control the seizure and abnormal discharge and avoid adverse reactions has always been the focus of research and attention of experts and scholars at home and abroad. With more and more literature reports and the promotion of continuous EEG monitoring technology, the understanding of EEG discharge mode of SE/RSE is changing rapidly. For generalized convulsive status epilepticus, if the clinical seizure symptoms disappear after anticonvulsant treatment, it does not mean that the patient's treatment is effective. If the patient's state of consciousness continues to not recover, there is often nonconvulsive status epilepticus (NCSE). Even accompanied by periodic waves [9], if such abnormal discharge is not found at this time, it can lead to continuous brain injury.

Levetiracetam, as a newly developed new antiepileptic drug (piracetam derivatives), has good pharmacokinetic characteristics and nearly 100% bioavailability. It is clinically used in the treatment of various states of epilepsy, such as convulsive epilepsy in children [10]. Synaptic vesicle protein SV2A in the brain is a unique site for its antiepileptic effect. SV2A is the binding site of levetiracetam in the brain, and levetiracetam plays an antiepileptic role by regulating the function of SV2A [11]. All products are excreted through the kidney, without pharmacokinetic interaction or respiratory inhibition, and can be applied to pregnant women (FDA: grade C) [12]. At present, benzodiazepines are mainly used for anticonvulsants, including fosphenytoin and valproate, and there are many relevant literature [13]. If levetiracetam injection can effectively control SE or even RSE, it may become a new type of intravenous drug in the field of antiepilepsy with the rapid effect, accurate efficacy, and few adverse reactions, which benefits patients a lot.

Since valproate is also widely used as a broad-spectrum antiepileptic drug in clinical practice, valproate and levetiracetam were, respectively, used in the treatment of epilepsy patients in this study, taking valproate as the control drug. This study focuses on the clinical therapeutic effect of levetiracetam compared with other second-line and third-line anticonvulsants in controlling epilepsy and abnormal EEG discharge.

## 2. Materials and Methods

### 2.1. Patients

In this study, patients with SE (including RSE) were collected from the Neurology Intensive Care Unit (NICU) of Qujing First People's Hospital. Admission criteria: patients who meet the diagnostic criteria of SE/RSE, including patients with NCSE and periodic epileptic discharge. Exclusion criteria: patients and their families refused to participate in this study, unable to cooperate with EEG monitoring, and patients in extremely critical condition or with endotracheal intubation. Informed consent was obtained from all patients, and informed consent was signed during the experiment. This study has been approved by the Ethics Committee of Qujing First People's Hospital.

### 2.2. Experimental Design

A prospective, parallel group design was used in this study. All patients in this study were diagnosed as SE. Before the experiment, general information and imaging examination data of patients were recorded, and continuous EEG monitoring was performed with brain function monitor; recording aEEG before using these drug experiments, patients were divided into 4 groups. According to relevant literature, the control group was injected with sodium valproate (Sichuan Keride Pharmaceutical Co., Ltd.); the first dose was 20 mg/kg intravenously, and the second dose was 1-2 mg/kg/d [14]. The experimental group was divided into 3 groups. The patients were injected intravenously with levetiracetam (registration number: H20170341) injection 500 mg/d, 1000 mg/d, and 1500 mg/d.

The contents of each group were as follows: when the patients had seizures, sodium valproate 1200 mg/d–1800 mg/d (according to bodyweight), 500 mg/d levetiracetam, 1000 mg/d levetiracetam, and 1500 mg/d levetiracetam were injected intravenously. After that, the patients who successfully controlled the symptoms were recorded, including the time of success, recurrence time, relapse patients with recurrence interval and adverse reactions, and abnormal EEG discharge.

### 2.3. Statistics and Analysis

In this experiment, excel 2013 software was used for data recording and SPSS17.0 software was used for data analysis. The probability of successful drug control of epilepsy, the probability of patient recurrence, the probability of abnormal EEG discharge, the average time taken for drug control of patient symptoms and the average time interval of patient recurrence were calculated. The ability of epilepsy control between the experimental group and the control group was compared. *T*-test was used to evaluate whether the difference of control success time and recurrence time between the experimental group and the control group was statistically significant. When *P* < 0.05, it is considered that the difference is significant.

## 3. Result

As given in Table 1, there were 60 patients in the sodium valproate control group, with a male-to-female ratio of 30/30 and an average age of 44 years. There were 34 patients with levetiracetam 500 mg/d. The male-to-female ratio was 18/16, and the average age was 38 years old. There were 54 patients with 1000 mg/d levetiracetam. The male-to-female ratio was 28/26, and the average age was 39 years old. There were 25 patients with levetiracetam 1500 mg/d. The male-to-female ratio was 15/10, and the average age was 36 years. The proportion of patients was similar, and there was no significant difference in the composition of causes. There was no significant difference in the composition of the four groups.

The experimental records of the patients after epileptic seizure are given in Table 2.

Compared with the sodium valproate control group, the treatment effect of the 1000 mg/d levetiracetam and 1500 mg/d levetiracetam groups in the experimental group was better, the success rate of controlling the symptoms of epilepsy was high, the time required to control the symptoms was short, the probability of recurrence was low, and the time required for recurrence was long.

The detection results of EEG are shown in Figure 1.  Figure 1(a) shows the EEG of the patient during the attack. Spike rhythm appears in most areas of the brain, and electrical interference is evident in the right guide muscle.  Figure 1(b) shows that the number of abnormal discharges decreased significantly after drug treatment.

There were some adverse reactions in the control group and levetiracetam 1500 mg/d and 1000 mg/d groups, and the difference was not statistically significant (P＞0.05). It is also worth noting that although the treatment effect of the 500 mg/d levetiracetam group was lower than that of the control group, none of the patients in the 500 mg/d levetiracetam group experienced adverse reactions compared to other groups and controls.

The experimental data were analyzed by SPSS 17.0 software. The results showed that there was no significant difference between the experimental group and the control group in the time required for symptom control by intravenous injection of levetiracetam 500 mg/d (*P* > 0.05), while the time required for symptom control by intravenous injection of levetiracetam 1000 mg/d and 1500 mg/d (*P* > 0.05). There were significant differences among the groups (*P* < 0.05). Analysis of the time interval between the second relapse and the first attack showed that there was no significant difference between the experimental group and the control group after intravenous infusion of 500 mg/d levetiracetam (*P* > 0.05), while there was a significant difference between the 1000 mg/d intravenous infusion of levetiracetam and the control group (*P* < 0.05).

## 4. Discussion

Epilepsy is one of the most common brain disorders in the world, affecting about 70 million people [14]. There are about 200 rare disorders that cause epilepsy [15]. However, the treatment of epilepsy is not satisfactory [16]. Ketogenic diet is a treatment for epilepsy in children, but it has obvious side effects, such as constipation and vomiting [17]. Besides, the anticonvulsant mechanism of ketogenic diet is still unclear, so research progress on epilepsy treatment drugs is still needed at present.

Levetiracetam is a new drug for the treatment of epilepsy, and there have been quite a number of studies to explore its application in the pediatric convulsive epileptic state of neonatal seizures [18]. In this study, the therapeutic effect of levetiracetam on SE and RSE compared with sodium valproate was explored. The effect of levetiracetam on abnormal EEG discharge was observed by electroencephalogram.

In this experiment, the proportion of male and female patients in the control group and the experimental group and the causes of epileptic seizures in patients with age were not significantly different, and absolute errors in patients were excluded as far as possible.

Our experimental results showed that compared with the control group of sodium valproate, the effect of high-dose levetiracetam on the treatment of epilepsy was faster than that of sodium valproate, and the effect was better. Moreover, the recurrence probability of patients in the high-dose levetiracetam group was significantly reduced, and the average recurrence time interval was very long, which indicated that the high-dose levetiracetam had a better effect in the treatment of epilepsy. In the analysis of the results of adverse reactions in patients, it was found that there was no statistically significant difference in the incidence of adverse reactions in several groups. While, the patients in the 500 mg/d levetiracetam experimental group did not have adverse reactions. Although in the experimental results of this study, patients in the experimental group of 500 mg/d levetiracetam had a poor treatment effect and a high recurrence rate, and the side effects of 500 mg/d levetiracetam on patients were also small, which may be an advantageous choice for some patients.

The detection results of abnormal EEG discharge show that the probability of abnormal EEG discharge in the experimental group of 1000 mg/d levetiracetam and 1500 mg/d levetiracetam is lower than that in the control group. After treatment with levetiracetam, although there were still some abnormal discharges, the frequency was significantly reduced, the attack time was shortened, and the patient's consciousness recovered. This shows that levetiracetam has a certain therapeutic effect in patients with abnormal EEG discharge. In this trial, this study found that the application of EEG technology can help us intuitively evaluate the changes of EEG in patients and combine with the clinical symptoms of patients, which is conducive to the conduct of the trial.

In conclusion, levetiracetam is a good antiepileptic drug. Compared with sodium valproate, high concentration levetiracetam has fast action time, good effect, low recurrence probability, and can control abnormal EEG discharge. Low concentration levetiracetam treatment slightly reduced, but less adverse reactions, and can also be used in some special patients. This study proved the clinical application value of levetiracetam, and both high-dose and low-dose levetiracetam could achieve the desired therapeutic effect. However, this study still has some limitations, the treatment of levetiracetam and sodium valproate produced relatively high adverse reactions, and the treatment of levetiracetam did not have an advantage in adverse reactions. In the later stage, drug combination can be considered to reduce the incidence of adverse drug reactions while ensuring the efficacy of drugs. Our study also found that the application of EEG technology in antiepilepsy treatment can not only monitor epilepsy symptoms but also evaluate the treatment effect and can play a certain role in epilepsy treatment.

## Figures and Tables

**Figure 1:** In the process of epilepsy patients with video electroencephalogram (EEG) (a) episodes, the patient is on the right side of body rigidity. In EEG, the spike rhythm broke out in the left central region, parietal region, occipital region, and posterior temporal region, and the electrical interference of the right guide muscle was obvious. (b) The application of levetiracetam injection for 211 seconds shows a slow wave background in EEG, and abnormal discharge was still observed in the right conductions, the number of which was reduced.

**Table 1:** Composition and pathogenesis of each group.

Group	Cases	Gender composition	Average age/years	Acute intracranial infection/case	Traumatic brain injury/case	Cerebrovascular disease/case	Self-withdrawal and poor control/case	Autoimmune encephalitis/case	CJD/case
Sodium valproate control group	60	30/30	41	44 (73.3%)	2 (3.3%)	3 (5.0%)	9 (15%)	2 (3.3%)	0
500 mg/d levetiracetam	34	18/16	38	20 (58.8%)	1 (2.9%)	3 (8.8%)	8 (23.5%)	2 (5.8%)	0
1000 mg/d levetiracetam	54	28/26	39	35 (64.8%)	1 (1.8%)	6 (11.1%)	7 (12.9%)	3 (5.5%)	2 (3.7%)
1500 mg/d levetiracetam	25	15/10	36	14 (56.0%)	1 (4.0%)	2 (8.0%)	5 (20.0%)	2 (8.0%)	1 (4.0%)

**Table 2:** Treatment effect statistics in each group.

Group	Successful symptom control/case	Average real time of successful control/cases	Recurrence of symptoms/cases	Recurrence time/min	Adverse reaction/case	Abnormal EEG discharge/case
Sodium valproate control group	39 (65.0%)	124	16 (41.0%)	115	8 (13.3%)	26 (43.3%)
500 mg/d levetiracetam	18 (52.9%)	104	12 (66.6%)	153	0	18 (52.9%)
1000 mg/d levetiracetam	42 (77.7%) ^*∗*^	70 ^*∗*^	13 (30%) ^*∗*^	260 ^*∗*^	3 (7.2%)	14 (33.3%) ^*∗*^
1500 mg/d levetiracetam	20 (80.0%) ^*∗*^	83 ^*∗*^	4 (20%) ^*∗*^	204 ^*∗*^	6 (24%)	5 (20.0%) ^*∗*^

Compared with the control group, ^*∗*^*P* < 0.05.

## Data Availability

The datasets used and/or analyzed during the current study are available from the corresponding author upon request.
